# Radiation dose reduction at a price: the effectiveness of a male gonadal shield during helical CT scans

**DOI:** 10.1186/1471-2342-7-5

**Published:** 2007-03-16

**Authors:** Lawrence T Dauer, Kevin A Casciotta, Yusuf E Erdi, Lawrence N Rothenberg

**Affiliations:** 1 Department of Medical Physics, Memorial Sloan-Kettering Cancer Center, 1275 York Ave. New York, NY 10021, USA

## Abstract

**Background:**

It is estimated that 60 million computed tomography (CT) scans were performed during 2006, with approximately 11% of those performed on children age 0–15 years. Various types of gonadal shielding have been evaluated for reducing exposure to the gonads. The purpose of this study was to quantify the radiation dose reduction to the gonads and its effect on image quality when a wrap-around male pediatric gonad shield was used during CT scanning. This information is obtained to assist the attending radiologist in the decision to utilize such male gonadal shields in pediatric imaging practice.

**Methods:**

The dose reduction to the gonads was measured for both direct radiation and for indirect scattered radiation from the abdomen. A 6 cm^3 ^ion chamber (Model 10X5-6, Radcal Corporation, Monrovia, CA) was placed on a Humanoid real bone pelvic phantom at a position of the male gonads. When exposure measurements with shielding were made, a 1 mm lead wrap-around gonadal shield was placed around the ion chamber sensitive volume.

**Results:**

The use of the shields reduced scatter dose to the gonads by a factor of about 2 with no appreciable loss of image quality. The shields reduced the direct beam dose by a factor of about 35 at the expense of extremely poor CT image quality due to severe streak artifacts.

**Conclusion:**

Images in the direct exposure case are not useful due to these severe artifacts and the difficulties in positioning these shields on patients in the scatter exposure case may not be warranted by the small absolute reduction in scatter dose unless it is expected that the patient will be subjected to numerous future CT scans.

## Background

The use of computed tomography (CT) scanning has increased rapidly since its introduction in the early 1970s. During the 1990s CT usage almost doubled, representing about 11% of radiology procedures in 1999 [1]. These values are consistent with a United States estimated rate for CT of 91 per 1000 population through the year 2000 [2]. In 1999, about 11% of all CT scans were performed on children age 0–15 years [1]. It is expected that the use of the modality will increase as the number of detectors and the clinical utility of CT is increased. It has been estimated that the number of CT scans performed annually has steadily increased in the U.S. from 2.8 million in 1981 [3] to 20 million in 1995 [2] and 60 million in 2006 [4], a number that seems destined to grow substantially. When using different sized acrylic phantoms to represent a range of pediatric and adult sizes undergoing CT with a typical 120 kVp x-ray beam, doses to the adult body range from 15–35 mGy while doses to the pediatric body are higher at 29–68 mGy using adult technique factors (milliampere-seconds)[5]. Similarly measured CT doses to the adult head range from 60–115 mGy while doses to the pediatric head are about 30% higher at 78–152 mGy using adult technique factors [5]. Also, when you have similar techniques, the effective doses are substantially higher in children by a factor of about 2 to 4 [6].

Simple dose reduction methods that do not impair diagnostic image quality should be considered for clinical use [7] in an effort to reduce risks of induced cancers and other effects [8]. Various authors have suggested that pediatric CT doses could be reduced by 30–50% or, more relative to adult doses, primarily by reducing the milliampere-seconds utilized, with no loss of diagnostic accuracy [5,9-14]. In a further attempt at reducing exposures to specific areas of the pediatric body, physicians are increasingly considering the use of shielding devices, including specially designed gonadal shielding for male testes. CT represents a shielding challenge because of the confounding dose from both the primary x-ray beam and the significant scatter component in the body during the multi-slice scanning.

The current approved recommendations by the International Commission on Radiological Protection suggests that the weighting factor for the male gonads is 0.20 based on the radiation sensitivity of the gonads due to the risk of mutagenesis [15], with the dose to the gonads therefore contributing 20% of the effective whole-body dose (note that the most recent draft recommendations suggest a reduced weighting factor of 0.08 for the gonads [16]). Various shielding designs have been developed over the years to reduce gonadal doses including lead blankets, bismuth shielding, clam-shell style male testicular shields, and flexible shields.

The goal of our phantom study was obtain information to assist the attending radiologist in the decision to utilize such male gonadal shields in pediatric imaging practice. Although previous studies have evaluated various male gonad shielding designs, we set out to measure the effect of a specific design made up of a 1 mm lead equivalent, flexible, velcro-held, wrap-around pediatric male gonad shield (Flexible gonad protector, Dr. Goos-Suprema, Heidelberg, Germany) on the testicular radiation exposure from both the primary beam and the scatter component during abdominal and pelvic helical CT scans using techniques utilized at our institution. In addition, the effect of the presence of the shield on the CT image was also evaluated.

## Methods

The study was performed using a sectional pelvic phantom (pelvic real-bone sectional phantom, Humanoid Systems – currently Radiology Support Devices, Inc., Long Beach CA, USA) (Figure 1), and as such, institutional review board approval was not required since no testing was performed on human subjects. The phantom consists of an adult male human skeleton embedded in tissue simulating plastic [17,18]. It is designed to simulate an average large (e.g. teen) pediatric or small adult patient's interaction with x-rays over the diagnostic energy range. No simulated organs exist within the phantom itself. A 6 cm^3 ^ion chamber (Model 10X5-6, Radcal Corporation, Monrovia, CA, USA) was placed on the phantom at the position of the male gonads (approximately 5 cm below the symphysis pubis and centered between the upper thighs) to measure the exposure in Roentgens (R) at this location (Figure 2). For the measurement and techniques employed, it was assumed that 1 Gy_tissue _≈ 1R × 0.91 (Gy_tissue_/R) [19].

When shielded exposure measurements were made, a 1 mm lead wrap-around gonadal shield (Figure 3) was placed around the ion chamber sensitive volume. As such, the ion chamber itself represented the gonads. The absence of testicular tissue equivalent material will have a minimal effect on results because it is expected that the significant majority of the scatter component is propagated from the body and pelvic bone tissues. The study geometry mimics the expected use of the shield during clinical applications

Two trials were evaluated. In the first trial, abdomen scans were performed to examine the effect of the shielding on scattered radiation only. For this abdominal scan trial, the ion chamber representing the testes, and the gonad shield were specifically placed approximately 5–10 cm outside of the scanning range so that the measured exposure represented only the scatter component. The abdomen of the phantom was scanned for this first trial using a routine abdominal examination protocol (Table 1, CT technique factors) on a 16 slice CT scanner (Lightspeed 16, General Electric, Waukesha, WI, USA) in a craniocaudal direction starting at a location just above the diaphragm and ending just above the bottom edge of the symphysis. The resulting scatter exposure was measured both with and without the gonadal shield in place. Because of limited access to the CT scanner, measurements using the large shield (650 cm^3^) were able to be repeated five times and only one measurement each were made using the small (150 cm^3^) and medium (450 cm^3^) shields.

In the second trial, a pelvis scan was performed to examine the effect of shielding on direct radiation (both primary and exit). In this trial, the pelvis of the phantom was scanned using the same routine abdominopelvic examination protocol (Table 1) in a craniocaudal direction from the area just above the bottom edge of the symphysis to the upper thigh. The resulting exposure was measured both with and without the gonadal shield in place. For this trial, measurements were also repeated five times for the large shield and one time each for the small and medium shields.

For both trials, the radiation exposures to the testicular region with and without the wrap-around gonadal shielding were compared using the Student's *t *test. Statistical significance was set at a *p *value of less than 0.05.

During both trials, representative CT images were obtained in order to evaluate image quality on the basis of noise measurements and visual inspection of image artifacts with and without the gonadal shield in place.

## Results

Tables 2 and 3 summarize the results of the phantom measurements, listing the gonad exposures without shields and with the large, medium, or small gonad shield in place. For the first technique, employing an abdominal scan with scatter dose to the gonads, the average measured gonad exposure was 68.6 mR (~ 0.62 mGy) without the gonad shield and was reduced to 29.1, 33.2, and 39.8 mR when the large, medium, or small shields were used, respectively. The shields appear to reduce scatter exposure to the gonads from an abdominal CT scan by about a factor of 2 (Table 2), a value shown to be statistically significant (*t *= 86, *p *< 0.001) with an absolute reduction in exposure of about only 20–30 mR. For the second technique, employing a pelvic scan with direct exposure to the gonads, the average measured gonad exposure was 4806 mR (~ 43.7 mGy) without the gonad shield and was reduced to 137.2, 171.4, and 265.4 mR when the large, medium, or small shields were used, respectively. The shields appear to reduce the direct exposure to the gonads by about a factor of 35 (Table 3), a value shown to be statistically significant (*t *= 1141, *p *< 0.001).

Images of an abdominal region were evaluated both with (Figure 4(A)) and without (Figure 4(B)) the gonad shield in place to measure noise within the same region. Noise was identical for each image, with a standard deviation of 5.5 Hounsfield Units in the region of interest (i.e. with or without the shield). When images of the pelvic region were evaluated with the gonad shield in place, severe streaking and image degradation was noted, as shown in Figure 5.

## Discussion

For the abdominal scans without gonadal shielding, the scatter exposure component to the gonads represented about 1.5% of the exposure to the gonads during a direct pelvic scan without gonadal shielding. For the abdominal scan, the large wrap-around shields appear to reduce the scatter exposure to the gonads by about 58%. For the direct pelvis scan, the exposure to the gonads was much higher, at 4820+/-14 mR, and the large wrap-around shields provided a more substantial shielding effect, reducing the direct beam exposure to the gonads by about 97%.

Price, et al [20] have performed a similar study that utilized a male Alderson therapy phantom, a 1 mm lead rubber wrap-around gonad shield, and lithium borate thermoluminescent dosimeters to measure doses to a testes phantom modeled from a single-slice CT scan. They found that doses to the gonads could be reduced by about 77% for scans outside of the gonadal area. They also reported severely degraded images for direct pelvic scans. Hidajat et al. [21] used a male Alderson radiation therapy phantom and protected the testes with a 1 mm lead testicular capsule to obtain a 95% reduction in dose. Hohl et al. [7] measured the dose to the gonads for 66 men (34 with 1 mm lead capsule shields and 32 without shields) that underwent routine abdominopelvic multi-detector CT with a 16 slice machine by using lithium fluoride thermoluminescent dosimeters. They report an 87% reduction in dose to gonads during abdominal scans. Table 4 compares the results of these literature reports including type of study, scanning protocol, testicular dose and percent reduction. While the doses to the shielded gonads are consistent with the literature values, there are differences in overall percent reduction that are most likely related to shielding types, setup, CT parameters, x-ray beam spectrum, geometry, and/or measurement techniques.

Image quality does not appear to be significantly affected when the scanned area is well outside of the gonadal shield location as was the case of the abdominal scan (Figure 4). Image quality is significantly reduced when the shield is located within the scan volume itself as was the case of the pelvic scan (Figure 5). The severe streak artifacts, caused by the presence of lead in the shield, render the image diagnostically unusable for most CT studies [22]. Therefore, an understanding of patient positioning and shielding usage is necessary. Although performed for general radiology applications and not for CT directly, a number of studies have shown that useful dose reduction tools such as simple shields are not always used correctly, resulting in inadequate coverage of reproductive organs because the shield was not positioned correctly, or inappropriately shaped or sized devices were utilized [23-25].

It is important to note that while gonadal shields may help reduce the scattered exposure component, there are other simple techniques that can be explored to reduce overall radiation exposure to pediatric patients. Geleijns et al. suggest that adjusting techniques, such as reducing tube current, can achieve an equal dose reduction while yielding better image quality compared with the use of shielding [26]. In a jointly issued guideline, the National Cancer Institute and the Society for Pediatric Radiology suggest the following reduction techniques for pediatric patients [27]: (1) perform only necessary CT examinations; (2) adjust exposure parameters for pediatric CT based on child size, region scanned, organ systems scanned, and scan resolution; and (3) to minimize the CT examinations that use multiple scans obtained during different phases of contrast enhancement (multiphase examinations) especially for body (chest and abdomen) imaging. The US Food and Drug Administration has also released recommendations for reducing pediatric CT doses that include[28]: (1) optimizing CT settings; (2) reducing the number of multiple scans with contrast material; and (3) eliminating inappropriate referrals for CT.

## Conclusion

A Humanoid phantom and a 6 cm^3 ^ion chamber can be very useful when performing shielding evaluation studies for CT scanning. The 1 mm wrap-around lead design for the gonadal shields reduced the already low scatter exposure to the testes by a factor of about only 2 with no appreciable loss of image quality. The shields reduced the direct beam exposure by a factor of about 35 at the expense of extremely poor image quality due to severe streak artifacts. Images in the direct exposure case are not useful due to these severe artifacts and the difficulties in positioning these shields on patients in the scatter exposure case may not be warranted by the small absolute reduction in scatter dose unless it is expected that the patient will be subjected to numerous future CT scans.

## Competing interests

The author(s) declare that they have no competing interests.

## Authors' contributions

LD and LR conceived of the study, collected the bulk of the data, and drafted the manuscript. KC and YE participated in the design and coordination of the study and assisted in the collection of the data. All authors read and approved the final manuscript.

## Pre-publication history

The pre-publication history for this paper can be accessed here:



## Figures and Tables

**Figure 1:** Humanoid abdominal/pelvic phantom.

**Figure 2:** **CT image of Humanoid phantom showing the location of the ion chamber at the level of the pelvis**. Ion chamber was located to approximate male gonad geometry (window level set at maximum to enhance the view of the chamber).

**Figure 3:** **1 mm lead wrap-around gonad shields in three sizes**. Flexible gonad protector, Dr. Goos-Suprema, Heidelberg, Germany.

**Figure 4:** **Comparison of abdominal CT images. **Abdominal CT images of Humanoid phantom both (A) with and (B) without the gonad shield in place. An identical region of interest (ROI), as indicated by the circle, was selected on each image to measure noise.

**Figure 5:** **Pelvic CT image of Humanoid phantom. **Pelvic CT image with gonad shield in place and directly situated in the beam. Note the severe streaking artifacts and general image degradation.

**Table 1:** CT technique factors utilized in this study

*Parameter*	*Value*
Technique	Adult – Helical
kVp	120
mA	260
Time per rotation (s)	0.7
mAs_eff_	194
Scan Field of View	Large
Z-axis collimation (mm)	1.25
Table speed (mm/rot)	18.75
Pitch	0.938
Reconstructed Scan Width (mm)	5

**Table 2:** Measured ion chamber readings (mR) representing gonadal exposure from an abdominal CT scan

*Scan #*	*No Shield*	*Large Shield (650 cm*^3^*)*	*Medium Shield (450 cm*^3^*)*	*Small Shield (150 cm*^3^*)*
1	69.7	29.4	33.2	49.8
2	68.7	29.5		
3	68.9	28.3		
4	68.3	29.0		
5	67.2	29.2		
Average +/- std.dev.	68.6 +/- 0.9	29.1 +/- 0.5		
% Reduction		58%	52%	42%
Reduction Factor		2.4	2.1	1.7

**Table 3:** Measured ion chamber readings (mR) representing gonadal exposure from a pelvic CT scan

*Scan #*	*No Shield*	*Large Shield (650 cm*^3^*)*	*Medium Shield (450 cm*^3^*)*	*Small Shield (150 cm*^3^*)*
1	4820	138.2	171.4	265.4
2	4800	138.3		
3	4800	138.9		
4	4810	136.4		
5	4800	134.2		
Average +/- std.dev.	4806 +/- 8.9	137.2 +/- 1.9		
% Reduction		97%	96%	94%
Reduction Factor		35	28	18

**Table 4:** Comparison of literature reports and present study for scattered dose reduction with the use of gonadal shields during abdominal CT scans (with the testes not in the direct beam)

*Study*	*Study Type*	*Scanning Protocol*	*Testicular Dose (mGy)*		*% Reduction*
				
			Without Shield	With Shield	
Hidajat et al. 1996 [19]	Phantom, 1 mm capsule	Single-slice sequential, 10 mm slice, 250 mAs/slice, 120 kV	1.46	0.07	95
Price et al. 1995 [18]	Phantom, 1 mm wrap-around lead rubber	Single-slice spiral, 10 mm slice, 220 mA, 120 kV	0.82^1^	0.19^1^	77
Hohl et al. 2005 [7]	Patient, 1 mm capsule	16-slice spiral, 16 × 1.5 mm collimation,150 mAs_eff_,120 kV	2.40	0.32	87
Present study	Phantom, 1 mm wrap-around canvas	16-slice spiral, 16 × 1.25 mm collimation 194 mAs_eff_, 120 kV	0.62	0.26	58

^1^Values initially reported in mSv and were converted to mGy for comparison, assuming 1 mSv = 1 mGy.
